This article has been retracted.

# Research on Piano Performance Optimization Based on Big Data and BP Neural Network Technology

**DOI:** 10.1155/2022/1268303

**Published:** 2022-02-22

**Authors:** Xueying Liu

**Affiliations:** Cai Jikun Conservatory of Music, Minjiang University, Fuzhou, Fujian Province 350108, China

## Abstract

At present, there are many chess styles in piano education, but there is a lack of comprehensive, scientific, and guiding teaching mode. It highlights many educational problems and cannot meet the development requirements of piano education at this stage. However, the piano scoring system can partially replace teachers' guidance to piano players. This paper extracts the signal characteristics of playing music, establishes the piano performance scoring model using Big Data and BP neural network technology, and selects famous works to test the effect of the scoring system. The results show that the model can test whether the piano works fairly. It can effectively evaluate the player's performance level and accurately score each piece of music. This not only provides a reference for the player to improve the music level but also provides a new idea for the research results and the application of new technology in music teaching. This paper puts forward reasonable solutions to the problems existing in piano education at the present stage, which is helpful to cultivate high-quality piano talents. Experiments show that the application of Big Data technology and BP neural network to optimize the piano performance scoring system is effective and can score piano music accurately. This paper studies the performance scoring system and gets the model after training, which can replace music teachers and alleviate the shortage of music teachers in the market.

## 1. Introduction

In recent decades, Chinese people's material life has seen abundant growth with the rapid economic development, and their aspiration for better spiritual life has been increasing and has become urgent. Therefore, more people choose to learn musical instruments, especially, piano. Nowadays, most piano learners are teenagers. One in every five families will send their children to learn piano performance, thus increasing the number of piano grading examinees year by year. However, the number of professional piano teachers is limited, so teachers become scarce resources, and due to the long-time neglect of art education in China, the imbalance of supply and demand has become more serious.

Big Data technology refers to the application of Big Data to the technological problems' solution. Big Data refers to data sets that are too large in scale to access, store, manage, and analyze with the traditional database software tools, featured by massive data size, rapid data flow, various data types, and low-value density [1, 2]. BPNN (back propagation neural network) is proposed by Rumelhart and McClelland et al., in 1986, which is a multilayer feed-forward NN (neural network) trained by error BP (back propagation) algorithm, and it has become the most widely used NN at present [3, 4].

BPNN is considered to be the most commonly used prediction method. The general structure of BPNN model is shown in the figure below. It is composed of input layer, hidden layer, and output layer, in which the hidden layer transmits important information between input layer and output layer. BPNN is the most basic neural network. Its output results adopt forward propagation, and the error adopts back propagation. BPNN has the function of supervised learning. Under the background of Big Data, the piano performance scoring system is built using the BPNN technology. First, in the introduction, the situation of the piano education market in China is introduced. Second, in the related works, the previous research is reviewed. Furthermore, in the method part, a scoring model based on Big Data and BPNN technology is constructed. Then, the test results of the proposed scoring model are discussed in the result section. Finally, the conclusion is summarized. The innovation here is to optimize the traditional NN model through the combination of Big Data technology and the BPNN model and to use the most appropriate algorithm to establish a performance evaluation model so that the performance evaluation of each piece of music is more accurate and sufficient. The research results provide a new perspective for computer technology to promote people's work and life.

This paper extracts the signal characteristics of playing music, establishes the piano performance scoring model using Big Data and BPNN technology, and selects famous works to test the effect of the scoring system. This paper is divided into five parts. The first part expounds the research background. At this stage, the development of piano education cannot meet the development requirements. However, the piano scoring system can partially replace teachers' guidance to piano players. In the second part, some references are cited to illustrate the extraction of signal characteristics of playing music and the establishment of piano performance scoring model using Big Data and BPNN technology. The third part establishes the piano performance scoring system and studies the functions of Big Data technology, BPNN technology, piano music feature extraction, performance scoring, and so on. In the fourth part, the performance of the scoring system is tested, and the notes, music bar score, and the whole music bar score are detected. Finally, the full text is summarized.

## 2. Related Works

In the context of Big Data, DL (deep learning) technology is widely used in all walks of life. At present, many experts and scholars have researched the application of DL technology. For example, Han et al. proposed an education development and evaluation model of intelligent learning environment, which integrated intelligent learning environment into learning ecology and education environment [5]. Liu et al. put forward an advanced regional cognitive ability training mode and applied DL in regional cognitive teaching through five teaching strategies: typical geographical real situation type, geographical depth problem type, interdisciplinary project type, emotion knowledge integration experience type, and field practice type of high-order thinking [6]. Maria et al. personalized online learning using Moodle in learning management systems, which improved students' academic performance and helped find students with difficulties [7]. Carin suggested a method using DL to integrate medical practice automation with medical education [8]. Ruhalahti et al. constructed the teacher's training assistance method using DL and inspired the thinking on the new development stage of designing and creating collaborative, self-management, and dialogue knowledge process [9]. Elbir et al. established a music scoring and recommendation model based on NN technology, which described music and score music with vectors [10]. Liu et al. proposed a combined algorithm for dam deformation prediction based on two traditional models and an optimized model, which combined two subalgorithms: GM (Grey Model) (1, 1) and BPNN [11]. Dekel et al. built the statistical basis and performance analysis of a new scoring system based on Naive Bayes classifier and 11-item validation questionnaires to test pain level [12]. Huang et al. suggested three different performance evaluation models: (a) a CNN (convolutional neural network) model using a simple time-series input, including aligned pitch contour and score. (b) A joint embedding model that could learn joint potential space of pitch contour and score. (c) A CNN model based on distance matrix, and the model of distance matrix between pitch contour and the score could predict the evaluation level [13]. He proposed a vocal music teaching system to automatically determine the level of piano players. The algorithm flow of the system was designed in detail with the principle of NN technology. The performance features of vocal music were extracted using Fourier transform and its improved function, and the key modules of the system were designed according to the system framework and data processing flow [14]. Chen et al. studied the application of DL in environmental monitoring and built a DL model for air pollution prediction using BPNN [15]. To sum up, Big Data, NN technology, and DL technology are used in all walks of life, especially, in education, which can alleviate teachers' burden by partly replacing their works.

The aforementioned research of Big Data technology and BPNN technology in different fields has proven that the related algorithms have been much matured and can be used in piano performance scoring systems. Meanwhile, different types of CNN result in different data accuracy. Here, the BPNN model is optimized, combined with Big Data technology, to make the scoring system model more effective.

## 3. Construction of Piano Performance Scoring System

### 3.1. Big Data Technology

Big Data refers to the data set that cannot be captured, managed, and processed by conventional software tools within a period. It is a massive, highly growing, and diversified information asset that needs a new processing mode to have stronger decision-making power, insight, and process optimization ability.

The biggest feature of Big Data is the huge amount of data. Traditional data processing software, such as Excel and MySQL, cannot analyze data well. Thus, the technology used in Big Data for data storage, processing, and calculation is completely different, such as Hadoop and Spark. Within the enterprise, the process of data production, storage, analysis, and application are interrelated, thus forming an overall Big Data architecture [16]. The basic architecture of Big Data is shown in Figure 1.

Generally, for Big Data technology, before the final view of data report or the use of data for algorithm prediction, data will go through the following processing steps [17].

- Data collection: it means to synchronize the data and logs generated by the application programs to the Big Data system.
- Data storage: massive data, which need to be stored in the system to facilitate the next use of the query.
- Data processing: the original data should be filtered, spliced, and converted at different levels before they can be finally applied. Data processing is a general term of these processes. Generally, there are two types of data processing: off-line batch processing and real-time online analysis.
- Data application: the processed data can provide external services, such as visual reports, interactive analysis, and training models for recommendation systems.

Here, the training set and test set are constructed for the model through Big Data technology.

### 3.2. BPNN Technology

#### 3.2.1. Deep Learning

The year 2006 has seen the appearance of a new research direction, DL, in the research field of ML (machine learning), which has been studied by academia and gradually applied by industry [18]. In 2012, Stanford University first builds a training model called DNN (deep neural networks) with a 16,000 CPU core parallel computing platform, which has made a great breakthrough in the application field of speech and image recognition [19]. In 2016, alpha dog, an artificial go software developed based on DL, defeats Li Shishi, the world's top go, master. After that, many well-known high-tech companies in the world begin to invest in DL technology, establish research institutes, and usher technical and R&D personnel into the field of DL.

ML technology studies how the computer simulates or realizes the learning behavior of animals, then learns new knowledge or skills, rewrites the existing data structure, and improves the program performance. Statistically, it is to predict the distribution of data, learn a model from the data, and then predict new data using this model. This requires that the test data and training data must be the same distribution. Its basic feature is trying to imitate the mode of information transmission and processing between neurons in the brain. The most significant applications are in the field of computer vision and NLP (natural language processing). Noticeably, DL is strongly related to NN in ML, and NN is also its main algorithm and means. In other words, DL is an improved NN algorithm. DL is divided into CNNs (convolutional neural networks) and DBNs (deep belief networks) [20]. Its main idea is to simulate human neurons. Each neuron receives information and transmits it to all adjacent neurons after processing.

#### 3.2.2. Artificial Neuron

An artificial neuron is a mathematical model created by imitating the basic operation function of a biological neuron, which has specific functions of a biological neuron [21]. The artificial neuron receives the given signal from the front neuron, and each given signal will be attached with a weight. Under the joint action of all the weight states, the neuron will show a corresponding activation state [22], which can be represented by equation (1).

(1) $$\begin{array}{c} f\left(x\right)=\sum_{i=1}^{n}x_{i}w_{i}. \end{array}$$

In equation (1), *f*(*x*) represents the final output state, *x*_*i*_ denotes the input signal, and *w*_*i*_ stands for the corresponding weight of the input signal, totaling *n* groups.

When the neuron receives a specific input signal, a specific signal will be output, and each neuron has a corresponding threshold. If the sum of the inputs received by the neuron is greater than the threshold, its state changes into the active state, and when it is less than the threshold, it is in the inhibitory state. The transfer functions of the artificial neuron are as follows:

(a) The expression of the linear function is shown in equation (2).
  (2) $$\begin{array}{c} f\left(x\right)=kx. \end{array}$$
(b) The slope function is expressed as in equations (3) to (5).
  (3) $$\begin{array}{c} f\left(x\right)=\alpha \left(x\geq \theta \right), \end{array}$$
  (4) $$\begin{array}{c} f\left(x\right)=kx\left(-\theta <x<\theta \right), \end{array}$$
  (5) $$\begin{array}{c} f\left(x\right)=-\alpha \left(x\leq \theta \right). \end{array}$$

The expression of transition function is shown in equations (6) and (7).

(6) $$\begin{array}{c} f\left(x\right)=\alpha \left(x\geq \theta \right), \end{array}$$

(7) $$\begin{array}{c} f\left(x\right)=\beta \left(x\leq \theta \right). \end{array}$$

The Sigmoid function is expressed as in equation (8).

(8) $$\begin{array}{c} f\left(x\right)=a+\frac{b}{1+e^{-\text{d}x}}. \end{array}$$

The transfer function should be selected according to the specific application range. The linear function will amplify the output signal. The nonlinear ramp function can prevent the impact of network performance degradation. The S-type function is used in the hidden layer.

#### 3.2.3. BP Neuron

Similar to artificial neuron, BP neuron also contains weight and summation. Specifically, *x*_*i*_ represents the input value of the *i*th neuron, *w*_*ji*_ stands for the weight value of the connection between the *i*th neuron and the *j*th neuron, *b*_*j*_ indicates the threshold, *y*_*j*_ denotes the output of the neuron *j*, and *f*(*x*) is the transfer function [23].

The net output *S*_*j*_ of the neuron *j* is shown in equation (9).

(9) $$\begin{array}{c} S_{j}=\sum_{i=1}^{n}w_{ji}\cdot x_{i}+b_{j}. \end{array}$$

When the threshold value is 0, the net output *S*_*j*_ of neuron *j* is shown in equation (10).

(10) $$\begin{array}{c} S_{j}=\sum_{i=1}^{n}w_{ji}\cdot x_{i}. \end{array}$$

#### 3.2.4. BPNN

BPNN is a multilayer feed-forward NN, featured by signal forward transmission and error BP. In forward transmission, the input signal is processed layer by layer from the input layer through the hidden layer to the output layer. The state of neurons in each layer only affects the state of neurons in the next layer. If the output layer cannot get the expected output, it will turn to BP and adjust the network weight and threshold according to the prediction error, so that the BPNN prediction output will continue to approach the expected output. BPNN must be trained before prediction to have associative memory and prediction ability. The training steps are as follows: (a) network initialization, (b) hidden-layer output calculation, (c) output-layer output calculation, (d) input-layer output calculation, (e) error calculation, (f) weight update, and (g) algorithm iteration is checked, and if the iteration is completed, the iteration continues, if not, steps (b) to (g) are repeated.

The BPNN algorithm is divided into two stages: the forward-propagation process and the BP process. In the process of forwarding propagation, the signal first comes from the input layer, passes through the hidden layer, arrives at the output layer, and then comes out from the output layer. Each layer of neurons can only affect the next state. When the output layer cannot receive the desired output correctly, it will use the BP process. Through the alternating operation of the two processes, the minimum value of the network error function will be found, and the operation of the NN memory will be completed [24].

The expression of the propagation process is shown in equations (11) and (12), in which equations (11) and (12) represent the outputs of the hidden layer and the output layer node, respectively.

(11) $$\begin{array}{c} z_{k}=f_{1}\left(\sum_{i=0}^{n}v_{ki}x_{i}\right),\;\left(k=1,2,\ldots ,q\right), \end{array}$$

(12) $$\begin{array}{c} y_{j}=f_{2}\left(\sum_{i=0}^{n}w_{jk}z_{k}\right),\;\left(j=1,2,\ldots ,m\right). \end{array}$$

In equations (11) and (12), *n* is the number of nodes in the output layer, *q* represents the number of hidden nodes, and *m* stands for the number of output layer nodes. *v*_*ki*_ indicates the weight of the connection between the input layer and hidden layer, *w*_*jk*_ represents the weight of the connection between output layer and hidden layer, *f*_1_(*x*) represents the transmission function of the hidden layer, and *f*_2_(*x*) stands for the transmission function of the output layer.

### 3.3. The Feature Extraction of Piano Music

The audio feature can show the MFCC feature of the *j*th music with the application *M*_*j*_, and the application *C*_*j*_ shows the Chroma feature of this work. Then, the notes can be quantified through the embedded technology, and then they are pretrained with FastText, so the word vector *v* is generated. Then, the vector of a single note in the song is multiplied by its own TF-IDF (term frequency-inverse document frequency) value, and the sum is averaged. Consequently, the lyrics feature vector is extracted for a music work [25].

TF-IDF value can indicate the importance of a phrase to its document. The importance of this phrase is directly proportional to its TF (term frequency) but inversely proportional to its IDF (inverse document frequency). The number of phrases is normalized using equation (13).

(13) $$\begin{array}{c} tf_{ij}=\frac{n_{ij}}{\sum_{k}nk_{j}}. \end{array}$$

In equation (13), *t*_*i*_ represents the phrase, *d*_*j*_ stands for the file, *tf*_*ij*_ denotes the above-IDF, *n*_*ij*_ indicates the number of times phrase *t*_*i*_ used in the data file *d*_*j*_, and ∑_*k*_*nk*_*j*_ represents the total number of phrases used in the file *d*_*j*_.

The IDF represents the importance of a note *idf*_*i*_ and is calculated through equation (14).

(14) $$\begin{array}{c} idf_{i}=\log\frac{\left|D\right|}{\left|D:i\right|+1}, \end{array}$$

|*D*| represents the total number of data files in the database, and |*D* : *i*| denotes the number of files with this note.

Equation (15) shows the value *tf*_*i*_*df*_*ij*_ of the phrase *t*_*j*_ in the file *d*_*j*_, and the important notes to the file can be obtained through filtering.

(15) $$\begin{array}{c} tf_{i}df_{ij}=tf_{ij}\times idf_{ij}. \end{array}$$

The eigenvector of the note is expressed as in equation (16).

(16) $$\begin{array}{c} L_{j}=\frac{\sum_{i}tf_{i}df_{ij}\times v_{i}}{\left|d_{j}\right|}. \end{array}$$

In equation (16), |*d*_*j*_| represents the number of notes in the phrase.

Figure 2 illustrates that the item side automatic encoder is used as the scoring model. MFCC feature *M*_*j*_, chroma feature *C*_*j*_, and lyrics feature *L*_*j*_ are applied to the input of the convolutional coding layer. The first layer is the convolution layer, the input is the two-dimensional feature *M* and *C*. Here, *X* denotes the input, and the input is equivalent to the feature map with two channels. *∗* represents the two-dimensional convolution operation that acts on the activation function and compresses the convolution input through a 2 × 2 pooling layer using an input of *K*1 convolution kernels and the weight of the first layer and outputs *A*^2^, with *K*1 channels. *A*^2^ is input into the second convolution layer, and *K*2 convolution kernels act on the activation function and outputs *A*^3^, with *K*2 channels. *A*^2^ and *A*^3^ are specifically expressed as in equations (17) and (18).

(17) $$\begin{array}{c} A^{2}=\text{pooling}\left(\sigma \left(\sum_{i}^{2}X_{i}*W_{i}^{1}+b^{1}\right)\right), \end{array}$$

(18) $$\begin{array}{c} A^{3}=\text{pooling}\left(\sigma \left(\sum_{i}^{K1}\overset{2}{\underset{i}{A}}*W_{i}^{2}+b^{2}\right)\right). \end{array}$$

The next part is the fully connected part of the automatic encoder, which is composed of a coding fully connected layer and a decoding fully connected layer. At the coding end, an additional connection layer is added, which makes the lyrics vector and the item side score vector in the scope network. The final coding vector *U* is represented as in equation (19).

(19) $$\begin{array}{c} U=\sigma \left(W^{3}A^{3}+V^{3}L+b^{3}\right). \end{array}$$

The later decoding end of the automatic encoder is opposite to this process, and the fully connected decoding end is expressed as in equations (20) and (21).

(20) $$\begin{array}{c} {\bar{A}}^{3}=\sigma \left({\bar{W}}^{3}U+{\bar{b}}^{3}1\right), \end{array}$$

(21) $$\begin{array}{c} \bar{L}=\sigma \left({\bar{V}}^{1}U+{\bar{b}}^{3}2\right). \end{array}$$

In equations (20) and (21), ${\bar{A}}_{3}$ and $\bar{L}$ corresponds to *A*^3^ and *L* in the encoder, respectively.

Then, the reverse of the convolutional coding layer is constructed, as shown in Figure 3, which is opposite to the convolutional coding layer and is represented by equations (22) and (23). The first is the upsampling layer, opposite to the pooling layer, which uses the nearest neighbor interpolation to double the dimension of ${\bar{A}}^{3}$. The second is the convolution layer with *K*1 convolution kernels, *∗* represents the two-dimensional convolution operation, and the output is ${\bar{A}}^{2}$. The third is the second upsampling layer, which doubles the input ${\bar{A}}^{2}$, uses two convolution kernels, and the outputs $\bar{X}$. Finally, the convolution layer with two convolution kernels, which convolutes the output ${\bar{A}}^{1}$ to the output $\bar{X}$. $\bar{X}$ represents two feature maps with the same dimension of two channels, corresponding to the reconstructed MFCC feature and Chroma feature, respectively.

(22) $$\begin{array}{c} {\bar{A}}^{2}=\sigma \left(\sum_{i}^{K1}\text{upsampling}\left({\bar{A}}^{3}\right)*{\bar{W}}_{i}{\;}^{2}+{\bar{b}}^{2}\right), \end{array}$$

(23) $$\begin{array}{c} {\bar{X}}^{2}=\sigma \left(\sum_{i}^{2}\text{upsampling}\left({\bar{A}}^{2}\right)*{\bar{W}}_{i}{\;}^{1}+{\bar{b}}^{1}\right). \end{array}$$

The stacked autoencoders are used for training, and the training process is as follows. After each pretraining, an additional layer is trained, and equation (24) is used as the overall loss function of the encoder.

(24) $$\begin{array}{c} L=\left(1-\alpha \right){\left(\bar{X}-X\right)}^{2}+\alpha {\left(\bar{L}-L\right)}^{2}+\lambda \left({\left\|W\right\|}^{2}+{\left\|M\right\|}^{2}+{\left\|N\right\|}^{2}\right). \end{array}$$

In equation (24), ${\left(\bar{X}-X\right)}^{2}$ represents the loss function of audio data, ${\left(\bar{X}-X\right)}^{2}$ denotes the loss function of music feature data, and ‖*W*‖^2^+‖*M*‖^2^+‖*N*‖^2^ stands for the regularization term. The parameter *α* indicates the weight represented by the item side score vector.

The degree of similarity influencing the results can be adjusted through *f*(*w*). Here, the exponential function *f*(*w*) is used for the experiment and is calculated as in equation (25).

(25) $$\begin{array}{c} f\left(w\right)=w^{q}. \end{array}$$

When the value *q* is higher in *f*(*w*), this model will focus on the impact most similar to the original musical works. When *q* = 0, this model will become a simple combination of scores.

### 3.4. Performance Scoring Function

The final scoring function is expressed as in equation (26).

(26) $$\begin{array}{c} h_{ui}^{U}=\sum_{v\in U}f\left(w_{uv}\right)r_{vi}=\sum_{v\in U\left(i\right)}f\left(w_{uv}\right). \end{array}$$

In equation (26), *h*_*u*_*i*__^*U*^ represents the score of the system for work *i* at the *u*th time, *w*_*uv*_ denotes the similarity between the original work and the music *uv* performed by the performer, *r*_*vi*_ stands for the score of the system for the *i*th work at the *v*th time, and *U*(*i*) is the overall data set. Hence, the user's score of the work is directly proportional to the similarity of the same track that the user has heard.

Combined with the calculation performance and its data, the item-based scoring function is improved, and equation (27) is obtained

(27) $$\begin{array}{c} h_{ui}^{S}=\sum_{j\in L}f\left(w_{ij}\right)r_{uj}=\sum_{j\in L\left(u\right)}f\left(w_{ij}\right). \end{array}$$

In equation (27), *h*_*u*_*i*__^*U*^ represents the system scoring of the work *i* for the *u*th time, and *w*_*ij*_ denotes the degree of similarity between works *ij*. In this scoring system, the similarity between music work *i* and the other work *j* recognized by the systems is proportional. *f*(*w*) is a monotone increasing function, which can strengthen or weaken the influence of similarity on the recommendation. The implied feature of a musical work is represented as *V*=(*V*_1_,…, *V*_*t*_), and *V*_*j*_ represents the implied feature vectors of the *j*th work, which express the characteristics of the work from different angles. After the results of *V* are obtained, *w*_*ij*_ is calculated as in equation (28).

(28) $$\begin{array}{c} w_{i}{\;}_{j}=\frac{V_{i}\cdot V_{j}}{\left|V_{i}\right|\left|V_{j}\right|}. \end{array}$$

The international standard for evaluating the correctness of multipitch detection is the *F*-measure index of note level. The larger the value is, the more effective the detection is. The calculation method is shown as in equations (29)–(31).

(29) Recall=nCorenRef,

(30) $$\begin{array}{c} \text{Precision}=\frac{n\text{Core}}{n\text{Tot}}, \end{array}$$

(31) F−measure=2Recall·PrecisionRecall+Precision.

In equations (29)–(31), *n*Core stands for the number of detected notes, *n*Re*f* denotes the total number of standard audio notes, *n*Tot represents the total number of detected notes, Recall indicates the relative detection accuracy of the score, and Precision is the relative detection accuracy of received notes.

### 3.5. Parameter Setting of BPNN

Here, a single-input neuron is used for the final comprehensive evaluation of the performance effect. In addition, to evaluate piano performance, two evaluation indexes: rhythm and expressiveness are needed. These two indexes also need two output neurons. Therefore, the output layer of the basic network structure needs three neurons. The previous output parameters need 60 neurons corresponding to the input layer, while the output layer needs three neurons. For the hidden-layer neurons, generally, only one hidden feed-forward NN is needed to approximate application functions in all cases. The structure and weight coefficient of BPNN should be determined through the learning method, thereby forming a correct mapping. The learning process of NN is to solve a group of weight coefficients with which the error function can reach the minimum under a specific network structure. Therefore, multiple groups of experiments are needed until a satisfactory model is obtained. Finally, 67 hidden layer nodes are determined.

The mean square error in the training process of the classical BPNN algorithm is expressed as in equation (32), the global error of the cumulative error BPNN algorithm is expressed as in equation (33), and the mean square error is expressed as in equation (34).

(32) $$\begin{array}{c} E_{p}=\frac{1}{2}\sum_{j=1}^{m}{\left(t_{j}^{P}-y_{j}^{P}\right)}^{2}, \end{array}$$

(33) $$\begin{array}{c} E_{p}=\frac{1}{2}\sum_{p=1}^{P}\sum_{j=1}^{m}{\left(t_{j}^{P}-y_{j}^{P}\right)}^{2}, \end{array}$$

(34) $$\begin{array}{c} \text{MSB}=\frac{1}{mp}\sum_{p=1}^{P}\sum_{j=1}^{m}\bar{{\left(y_{kj}-y_{kj}\right)}^{2}}. \end{array}$$

In equations (32) to (34), *E*_*p*_ represents the error, *t*_*j*_^*p*^ denotes the actual output of the *j*th time, and *y*_*j*_^*P*^ stands for the expected output of the *j*th time. *m* indicates the number of output nodes, *P* represents the number of training samples, *y*_*kj*_ denotes the actual output of BPNN, and $\bar{y_{kj}}$ stands for the expected output of BPNN.

## 4. Performance Test of the Scoring System

Sound can be regarded as waves in air, water, and other media. When we record sound, we record the pressure of the medium on the microphone, more precisely the wave amplitude. Digital recording goes further because it must discrete the recording process. The microphone is sampled at a very high frequency. The higher the frequency, the better the recording quality. This frequency is also called the sampling rate. The standard CD audio sampling rate is 44,100 Hz (Hertz). This means that we get 44,100 microphone amplitude measurements per second. In this case, the measurement is usually called sampling, and each sampling step returns us a so-called sample. The sample represents the amplitude measured by the microphone at a given time. The value of the sample must be stored in some way.

### 4.1. Detection of Musical Notes

Here, six pieces of music are tested by note-level test, bar score test, and whole score test. A, B, C, D, E, and F refer to each composition, respectively. A represents Blue Danube, B denotes Etude, C indicates Coming in February, D stands for Fugue, E is Nocturne, and F is Goddess Dance.

Figures 4 and 5 show the test index results and the final score of the note level evaluation of the six songs.

Figure 5 illustrates that the score index of composition F is the lowest, and the score index of composition A is the highest. Except for composition A, the final scores of other songs are all above 0.93, precision is above 0.91, and F-measure is above 0.93. This is because composition A is a world-class famous music, and its complexity is much larger than the other five pieces. Therefore, the note-level evaluation is good for the judgment of non-top music performance, which is much higher than 0.89 of the mainstream judgment methods.

### 4.2. Detection of Music Bar Score

This study tested the performance of six compositions by bar score. A, B, C, D, E, and F refer to each composition, respectively. The accuracy of bar performance in the test set is divided into four segments: less than 60%, 60% to 70%, 70% to 80%, and more than 80%. The actual, correct, and multidetection numbers are recorded. The detection rate is equal to the ratio of the number of correct detection and the actual number.

Figures 6 and 7 display the bar score test results and the final detection rate of the six compositions.

Figures 6 and 7 demonstrate that the detection rate of each composition is more than 93%, and the average detection rate of six compositions is 96.79%. After the scoring area is divided, most of the detection accuracy is between 82% and 93% because the accurately detected notes may not all be accurately converted into vector features, and inaccurate conversion leads to the decline of the subsequent detection rate.

### 4.3. Detection of the Score of the Whole Music

The performance of six pieces of music is tested by a whole score test. A, B, C, D, E, and F refer to each composition, respectively. Ten samples are selected for the comparison between the overall detection accuracy and the actual detection accuracy. The accuracy is equal to the ratio of the number of correct detection and the actual number.  Figure 8 shows the score test results of the six compositions, and Figure 9 illustrates the total deviation and average deviation of the score test.

Figure 9 implies that the average deviation of the whole score test of each sample is less than 5. The average deviation of the whole score test of composition A is the smallest, only 2, and the total deviation is only 20. The average deviation of composition C is the largest, reaching 3.5, and the total deviation is 35, which is 1.75 times that of music A. The performance test result of composition C is 98%, and the accuracy is 100%. The score deviation of composition A is not big, so the actual performance accuracy is 100%, and the score deviation of other compositions is also within 5%. Overall, the performance detection accuracy is more than 93%, so it is within a reasonable error range.

## 5. Conclusion

Here, a piano performance scoring system model is studied based on Big Data and BPNN technologies to replace music teachers and alleviate the short supply for music teachers in the market. First, Big Data technology is introduced and used to search the data training set and test set for piano performance scores. Then, the performance score system is constructed by BPNN technology, and all notes are transformed into corresponding feature vectors. Consequently, the performance score system is trained and the model is obtained. Finally, the experiment shows that the application of Big Data technology and BPNN in the optimization of the piano performance scoring system is effective and can accurately score piano music.

However, there are still some deficiencies in this paper. Although this study has achieved the expected research objectives and reached some valuable research conclusions, the compatibility of the model is insufficient. Owing to the inability to seek the help of first-class musicians, the model may not be able to accurately identify piano music. This also points out the direction for our future research. In the future, we will focus on the following two aspects: further improving the compatibility of the model and optimizing the code. Contact first-class pianists to understand the actual situation of piano performance and optimize the model.

## Figures and Tables

**Figure 1:** The basic architecture of Big Data.

**Figure 2:** Convolutional coding layer.

**Figure 3:** Convolutional decoding layer.

**Figure 4:** Test index results of note-level evaluation.

**Figure 5:** Final scores of note-level evaluation.

**Figure 6:** Bar score test result (a) above 80, (b) 70–80, (c) 60–70, (d) below 60.

**Figure 7:** Final detection rate.

**Figure 8:** Score test results of music.

**Figure 9:** Total deviation and average deviation in score test of the whole composition.

## Data Availability

The data used to support the findings of this study are available from the corresponding author upon request.
